# Down-regulation of siglec-2 (CD22) predicts worse overall survival from HBV-related early-stage hepatocellular carcinoma: a preliminary analysis from Gene Expression Omnibus

**DOI:** 10.1042/BSR20181423

**Published:** 2018-11-28

**Authors:** Xiaojing Ren, Yuanyuan Ji, Xuhua Jiang, Xun Qi

**Affiliations:** Department of Liver Disease, Shanghai Public Health Clinical Center, Fudan University, Shanghai 201508, China

**Keywords:** alpha-fetoprotein, hepatocellular carcinoma, overall survival, prognosis, siglec-2

## Abstract

Sialic-acid-binding immunoglobulin-like lectin (siglec) regulates cell death, anti-proliferative effects and mediates a variety of cellular activities. Little was known about the relationship between siglecs and hepatocellular carcinoma (HCC) prognosis. Siglec gene expression between tumor and non-tumor tissues were compared and correlated with overall survival (OS) from HCC patients in GSE14520 microarray expression profile. Siglec-1 to siglec-9 were all down-regulated in tumor tissues compared with those in non-tumor tissues in HCC patients (all *P* < 0.05). Univariate and multivariate Cox regression analysis revealed that siglec-2 overexpression could predict better OS (HR = 0.883, 95%CI = 0.806–0.966, *P* = 0.007). Patients with higher siglec-2 levels achieved longer OS months than those with lower siglec-2 levels in the Kaplan–Meier event analysis both in training and validation sets (*P* < 0.05). Alpha-fetoprotein (AFP) levels in siglec-2 low expression group were significantly higher than those in siglec-2 high expression group using Chi-square analysis (*P* = 0.043). In addition, both logistic regression analysis and ROC curve method showed that siglec-2 down-regulation in tumor tissues was significantly associated with AFP elevation over 300 ng/ml (*P* < 0.05). In conclusion, up-regulation of siglec-2 in tumor tissues could predict better OS in HCC patients. Mechanisms of siglec-2 in HCC development need further research.

## Introduction

Hepatocellular carcinoma (HCC) is the fifth most common cancer and the second most common cause of cancer-related deaths [1–3]. In the past two decades, a marked increase in HCC-related annual death rates was observed [2,4]. And, the incidence of HCC will continue to rise until 2030 based on a SEER registry projects study [5]. Previous research revealed that the prediction of prognosis plays a critical role in therapeutic options of HCC. But, little tumor markers have been externally validated in HCC survival prediction [6]. To find novel biomarkers for predicting HCC prognosis, and to reveal HCC target for treatment is urgently required.

As a characteristic of cancer, immune evasion is more prevalent in organs with high immune tolerance including the liver [7]. The sialic-acid-binding immunoglobulin-like lectins (siglecs), a novel family of immunoregulatory, have received more and more attention for their capacity to mediate cell death, anti-proliferative effects and to regulate a variety of cellular activities [8]. Currently, pharmacological strategies using siglec agonistic cross-linking therapeutics are discussed. Modulation of immune responses by targeting siglecs using agonistic or antagonistic therapeutics may have important clinical implications and may be a novel pharmacological strategy in tumor immunotherapy [8]. A recent research has revealed that high expression of siglec-10 on NK cells mediates impaired NK cell function, and siglec-10 expression in tumors is associated with poorer survival of HCC patients [9]. However, roles of siglec family in HCC development were little discussed.

According to the potential value of siglecs in HCC development, this study aimed to evaluate the associations between siglec family and outcomes from hepatitis B virus (HBV)-related HCC patients, hoping that the data may provide potential biomarker candidates and useful insights into the pathogenesis and progression of HCC.

## Materials and methods

### Patients

Using GSE14520 profile from Gene Expression Omnibus (GEO, http://www.ncbi.nlm.nih.gov/geo/) database, 247 patients with HCC were identified. Twenty-seven patients were excluded for the unavailable siglec gene expression or insufficient clinical outcome data. Finally, 220 HCC cases were included in the analysis. All the HCC patients had a history of HBV infection or HBV-related liver cirrhosis; the diagnosis of HCC was made in all cases by two independent pathologists who had detailed information on clinical presentation and pathological characteristics as declared by Roessler et al. [10].

All liver tissue was obtained with informed consent from patients who underwent radical resection between 2002 and 2003 at the Liver Cancer Institute and Zhongshan Hospital, Fudan University. The study was approved by the Institutional Review Board of the participating institutes [10]. All participants provided written informed consent, as reported by Roessler et al. [10,11].

### Data extraction and end points

We extracted the GSE14520 microarray expression profile. Tumor sample and microarray processing were reported by Roessler et al. [10,11] and are available at http://www.ncbi.nlm.nih.gov/geo/query/acc.cgi?acc=GSE14520. The experiment protocols and data processing methods are available at http://www.ncbi.nlm.nih.gov/geo/query/acc.cgi?acc=GSM362949. Siglec gene expression levels were calculated using the matchprobes package in the R program and the log2 RMA-calculated signal intensity was reported. Nine siglecs including siglec-1, siglec-2, siglec-3, siglec-4, siglec-5, siglec-6, siglec-7, siglec-8 and siglec-9 were searched and included in our analysis. Overall survival (OS) was defined as the time from surgery to death from any disease.

### Statistical analysis

PASW Statistics software version 22.0 from SPSS Inc. (Chicago, IL, USA) was used for statistical analysis. Student’s *t*-test, Mann–Whitney *U*-test and Chi-squared test were used for normally distributed continuous data, non-normally distributed continuous data and categorical variables, respectively. Univariate analysis and multivariate Cox and logistic regression were assessed for identifying factors associated with OS and clinico-pathological features. The Kaplan–Meier curve by log rank method was used to compare OS between different groups. A two-tailed *P* < 0.05 were considered statistically significant.

## Results

### Siglec levels comparison between tumor and non-tumor tissues

Nine members of siglec family were identified, including siglec-1 to siglec-9. As shown in Figure 1, all siglecs were overexpressed in non-tumor tissues compared with those in tumor tissues (all *P* < 0.05, Figure 1).

**Figure 1:** Differential expression of siglecs between non-tumor and tumor tissues in HCC patients

### Relationship between siglecs and HCC overall survival

As shown in Table 1, univariate analysis showed that siglec-2 and siglec-4 were potential factors associated with HCC OS (*P* = 0.065 and *P* = 0.061, respectively). When all siglecs were evaluated by a multivariate model using enter selection, up-regulation of siglec-2 in tumor tissues showed protective potentials for HCC OS (HR = 0.883, 95%CI = 0.806–0.966, *P* = 0.007). In contrast, siglec-4 overexpression was negatively associated with HCC OS (HR = 1.059, 95%CI = 1.025–1.094, *P* = 0.001).

**Table 1:** Univariate and multivariate Cox regression analysis of siglecs and HCC overall survival

Siglecs, per increase of 1 unit	Univariate analysis		Multivariate analysis	
	HR (95%CI)	*P* value	HR (95%CI)	*P* value
Siglec-1	0.988 (0.971–1.006)	0.18		
Siglec-2	0.932 (0.65–1.004)	0.065	0.883 (0.806–0.966)	0.007
Siglec-3	1.005 (0.979–1.032)	0.708		
Siglec-4	1.028 (0.999–1.058)	0.061	1.059 (1.025–1.094)	0.001
Siglec-5	1.025 (0.968–1.084)	0.397		
Siglec-6	0.995 (0.911–1.087)	0.917		
Siglec-7	1.003 (0.94–1.07)	0.939		
Siglec-8	1.018 (0.898–1.153)	0.783		
Siglec-9	1.004 (0.864–1.167)	0.957		

Furthermore, we performed *R* software analysis to determine the cut-off values of siglec-2 and siglec-4 for the prediction of OS in the training set. Then, we transformed the continuous data above into dichotomous variables according to the determined cut-off values. Unfortunately, no statistical significance was found between siglec-4 and HCC OS in training set based on randomized sampling. According to *R* language analysis, we grouped siglec-2 using cut-off values of 11.6 into siglec-2 low group and siglec-2 high group. This demonstrated that patients in siglec-2 high group had better OS than those in siglec-2 low group, both in training set and validation set (log rank *P* = 0.041 and log rank *P* = 0.031, respectively, Figure 2A,B). When all HCC patients were included in the Kaplan–Meier event analysis, patients with higher siglec-2 levels achieved longer OS months than those with lower siglec-2 levels (mean survival months in siglec-2 high group = 50.9 ± 1.8 and in siglec-2 low group = 41.5 ± 3.9, respectively, log rank *P* = 0.01, Figure 2C).

**Figure 2:** Association between siglec-2 expression and OS in HCC patients Higher siglec-2 levels are associated with better OS in HCC patients, in training set (**A**), validation set (**B**) and total database (**C**).

### Relationship between siglecs and HCC clinico-pathological features

We grouped HCC patients with siglec-2 cut-off of 11.6 and compared differences of clinico-pathological features between these two groups. As shown in Table 2, more patients had higher alpha-fetoprotein (AFP) levels in siglec-2 low group than those in siglec-2 high group (60% vs. 41.7%, *P* = 0.043). Additionally, no differences were found in patients’ clinico-pathological features including HBV virus status, ALT levels, tumor size, multinodular, cirrhosis and tumor staging (all *P* > 0.05).

**Table 2:** Clinico-pathological features based on siglec-2 expression in HCC patients

Clinico-pathological features	High siglec-2 group (*n* = 180)	Low siglec-2 group (*n* = 40)	*P* value
Gender (male/female), *n*	156/24	34/6	0.781
Age (>50 years/<50 years), *n*	99/81	25/15	0.387
HBV viral status (AVR-CC/no/NA), *n*	47/128/5	9/27/4	0.111
ALT (>50/<50/NA), U/l	76/104	14/26	0.401
Main tumor size (>5/<5/NA), cm	66/114/0	14/25/1	0.104
Multinodular (yes/no), *n*	37/143	7/33	0.662
Cirrhosis (yes/no), *n*	163/17	39/1	0.147
TNM staging (I–II/III/NA), *n*	138/40/2	31/8/1	0.763
BCLC staging (0-A/B-C/NA), *n*	138/41/1	30/9/1	0.503
CLIP staging (0/1/2/3/4/5/NA), *n*	81/61/25/8/2/1/2	15/13/9/1/1/0/1	–
AFP (>300/<300/NA), ng/ml	75/102/3	24/16/0	0.043

AFP, alpha-fetoprotein; ALT, alanine aminotransferase; AVR-CC, active viral replication chronic carrier; NA, not available.

We performed logistic regression analysis to identify the relationship between siglecs and HCC clinico-pathological features. This was summarized in Table 3. Univariate analysis showed that siglec-2 was a potential factor associated with AFP levels in HCC patients (*P* = 0.012). When all siglecs were evaluated by a multivariate model using enter selection, siglec-2 overexpression is negatively associated with HCC patients’ AFP level (OR = 0.822, 95%CI = 0.724–0.934, *P* = 0.003). To evaluate the predictive accuracy of siglec-2 and siglec-4 for AFP levels in HCC patients, we analyzed ROCs and found that elevated siglec-2 significantly and accurately predicted lower AFP level (AUC = 0.607, *P* = 0.007, Figure 3).

**Figure 3:** ROC curve of siglec-2 for AFP > 300 ng/ml

**Table 3:** Relationship between siglecs and HCC clinico-pathological characteristics by logistic regression analysis

Siglecs, per increase of 1 unit	AFP > 300 ng/ml			
	Univariate analysis		Multivariate analysis	
	OR (95%CI)	*P* value	OR (95%CI)	*P* value
Siglec-1	1.001 (0.984–1.018)	0.936		
Siglec-2	0.891 (0.815–0.975)	0.012	0.822 (0.724–0.934)	0.003
Siglec-3	1.0 (0.967–1.035)	0.992		
Siglec-4	1.034 (0.969–1.102)	0.313		
Siglec-5	1.028 (0.944–1.12)	0.523		
Siglec-6	1.045 (0.932–1.173)	0.449		
Siglec-7	1.044 (0.959–1.137)	0.316		
Siglec-8	1.063 (0.908–1.245)	0.448		
Siglec-9	0.861 (0.714–1.038)	0.117		

### Siglec-2 coexpression genes and pathways enrichment

Using the GSE14520 microarray database, coexpressed genes of siglec-2 in HCC were searched in HCC. As shown in Table 4, 137 genes were found to be positively coexpressed with siglec-2. On the other hand, 352 genes were negatively coexpressed with siglec-2 as shown in Table 5.

**Table 4:** Siglec-2 positive coexpressed genes (*n* = 137)

ACADS	TG	PLCB2	NNAT	LCAT	GNAO1	VIPR1	CD79A	GPR162	MYLPF
RIN1	ESR1	RCE1	SULT2B1	TCP11L1	MYOM2	CD33	LLGL1	WNT10B	PRKCG
ADCYAP1	NPHP1	ELAVL3	SCN2A	CACNG3	PDE3A	KLKB1	INSL4	F11	MYOD1
UMOD	CUBN	NAT2	ADRB3	NGF	STATH	IL11	HTR6	AKAP4	CHRND
LTK	SLC6A13	NOS1	KCNS1	POU6F2	CRYGD	SLC28A1	FOXH1	CRYBB3	CACNB4
PRMT8	CD160	SCN7A	BMP8B	MYBPC3	PSD	GIPR	OSBPL7	RASGRP2	BMP3
CYP2A13	GLP1R	SLC14A2	GJA8	EYA2	CORO2B	PDE6G	CHRNA3	NR6A1	CLEC4M
TACR1	GRIN1	ADRA1D	BMP7	DSCAM	TUBB7P	CAMK2A	SH3BP1	GPD1	MYOZ3
PRSS53	FSHB	GPR182	PLAC4	TOM1L2	EMX1	CFAP74	DNAH2	CFAP70	MYCNOS
CYP2A7P1	LOC101929073	DDR1-AS1	KLK1	LINC01482	GRIK5	FUT7	CNPY4	TTC38	ECHDC2
A4GALT	MYOZ1	NLGN3	CPLX3	SLC13A4	RNF122	RETN	CARD14	KCNQ1DN	NOX5
LINC00652	PLA2G3	THEG	CTNNA3	GABRQ	CHST8	GSN-AS1	C7orf69	CLDN17	HOXC8
ZNF717	FGF17	TAS2R7	IL36A	OR1D2	MYL10	LZTS1	CLEC4A	KIAA1644	LRCH4
DMWD	ADRBK1	PNPLA2	ACACB	CACNG4	LOC100505915	NPEPL1			

**Table 5:** Siglec-2 negative coexpressed genes (*n* = 352)

EIF4G2	RPS5	CBX3	ZNF146	ILF2	RPL30	RPL37	HNRNPU	NCL	CLTC	PTGES3	YWHAZ
PHB	DYNLL1	MAPRE1	CAPRIN1	RPS27	GNB1	RAN	HNRNPC	CALU	RPLP1	LAMC1	XRCC6
SNRPD2	ZNF207	CCT4	SSR1	CCT3	DEK	IPO7	ACTR3	YWHAH	EIF5B	RPS18	TUBA1B
ARF4	CSE1L	ACLY	SSB	UBA2	PSMD1	PCNA	CAPZA2	PSMC4	RPS16	SRP9	TOP2A
PPIA	CCT6A	UBE2D2	YME1L1	TPD52L2	PPP1CB	BUB3	VBP1	RRM1	RCN2	TOMM70A	CBX1
UBE2N	RPA1	TRIP12	MCM3	NME1	SEC23B	PPP4R1	ZC3H15	PWP1	ACP1	ITGA6	ARL1
SMC4	MARCKS	PSMC6	TUBG1	CDC123	WSB2	ADNP	VPS26A	NET1	HDAC2	RRM2	CKS1B
UBE2A	MCM6	CPD	CCT2	RSU1	KIF5B	MORF4L2	LANCL1	DPF2	PRPF4B	PPP1R2	VEZF1
NUP133	SRPK1	STT3A	EIF3M	PSMB4	CDK4	VPS72	STAG1	SMARCA5	ACBD3	UBE2K	PSMD12
USP1	CPSF6	H2AFV	KIAA0101	GMFB	HSPA13	TYMS	SSBP1	HTATSF1	TOPBP1	NRAS	LPGAT1
ACTL6A	GTF2A2	SNRPD1	UBE2S	PIGC	CDC20	SRSF3	HLTF	TXNDC9	DNM1L	HAT1	SRPK2
CDK1	MAPK9	HS2ST1	SNRPE	PPP2R5E	RBBP8	EZH2	PSMA4	MFAP1	SUCO	RPP30	SEC61G
STAM	PTTG1	CD2AP	RTCA	COIL	RFC2	UTP18	TRIP4	C5orf22	TDG	BUB1B	SNRPF
RFC4	ZWINT	CKS2	DBF4	CEP350	PPM1D	IARS	FEN1	EEF1E1	VRK2	HNRNPA2B1	SRP19
PFDN4	SNRPG	KIN	SLBP	GINS1	NUP155	MFN1	NIPBL	CAND1	NCKAP1	NUP62	RBM3
CLIC1	RPN2	RPS3	PRKDC	ARPC3	YWHAB	NAP1L1	HNRNPR	PSMD11	MRPL3	HMGB2	PTK2
POLE3	CANX	STK24	TXN	ILF3	PRCC	SEPHS1	BECN1	DNAJB6	ABI1	SF3B4	GLRX3
UFD1L	DR1	FAM208A	SWAP70	SLC35A2	POLR3C	BAG2	MSH2	EED	MRPL9	SOCS5	CHUK
PRKCI	CDKN3	PHTF2	HMGN4	CNPY2	UBE2E3	TPX2	NOL7	HSP90AA1	PSMD4	CACYBP	PDCD10
MCM7	HSPA4	CDK7	COX11	TUBA1C	KPNA2	HSPA5	ITGB1	SMARCE1	RPL7	U2SURP	LSM14A
RBM12	ANKLE2	NUP205	WAPL	SERPINB1	MAPK1	PSMD14	CLASP2	GNS	DESI2	KIAA0368	SNRNP27
AVL9	UBE2E1	NEK7	AQR	MAPK1IP1L	KDM3A	NUP160	ATF2	TRIM37	DNAJC9	SP3	SNRPB
RHEB	TUBB3	H2AFZ	HSP90AB1	GMPS	RALA	H2AFY	SUB1	RIF1	CCNB1	SNW1	SUMO4
CLTA	MIR1244-3	PDIA6	HN1	ALDH18A1	UFC1	ENAH	SYNCRIP	PRELID3B	CDC27	DYNLRB1	MRPL42
SAE1	CNOT6	MORF4L1	ASNSD1	PRC1	NUP85	NUSAP1	PRPF40A	AGFG1	MRPS10	ARMC1	GOLT1B
TMEM258	GTPBP4	MEX3C	CKAP2	MAP4K3	FAM208B	PFDN2	GMNN	RIOK2	MRS2	LYRM4	DUSP12
CDC73	DTL	HEATR1	NUP37	NXT1	IFT52	CNIH4	NUP107	RPAP3	PPP2R3C	RPS6KC1	TMEM106B
TPRKB	RRP15	HSPA14	TMEM185B	OLA1	PSMD10	UXS1	ECT2	UCHL5	SAP130	NAA35	ARID4B
LYRM2	TBL1XR1	ARPP19	ANP32E	DENR	MED17	PRPF18	METTL5	DDX50	ADSS	SEH1L	NOL11
PAPOLA	MCM4	RACGAP1	THOC2								

Additionally, gene set enrichment analysis (GSEA) was used for identification of putative KEGG pathways associated with siglec-2 coexpressed genes. Consequently, pathways including MAPK signaling pathway and calcium signaling pathway, which have been proved in liver cancer, were significantly enriched with siglec-2 positively coexpressed genes (*FDR* < 0.05, Figure 4), While siglec-2 with its negatively coexpressed genes contributed to tumor cell phenotype including cell cycle, spliceosome, DNA replication, ubiquitin-mediated proteolysis, proteasome, oocyte meiosis, mismatch repair, ribosome, pathways in cancer and pathogenic *Escherichia coli* infection (*FDR* < 0.05, Figure 5).

**Figure 4:** KEGG functional enrichment of siglec-2 with its positive coexpressed genes

**Figure 5:** KEGG functional enrichment of siglec-2 with its negative coexpressed genes

## Discussion

Immunotherapy for HCC has shown some success [7]. However, in most HCC patients or animal models, tumors progressed in spite of tumor-specific immune responses [12]. Thus, to find new immune markers of HCC development is still of significant importance. Functionally, siglecs participate in regulating the innate and adaptive immune responses through the recognition of their glycan ligands [13]. They have been demonstrated to be involved in a series of inhibitory processes, cell–cell interaction processes and endocytosis [8,14–16]. In our analysis, we found that all siglecs including siglec-1 to siglec-9 were significantly suppressed in HCC tumors, which may serve as anti-oncogenes. Recently, several studies revealed that siglec deficiencies contributed to the potential for generation of malignancy like lymphomas and leukemias [17,18]. As reviewed by Macauley et al., siglecs played a role in regulating of immune surveillance of cancer by keeping with their roles aiding immune cells in distinguishing between self and non-self [13]. They concluded that siglecs effectively reduce innate immune responses against cancer cells by down-regulating immune cells that express them through recognition of sialoside ligands on the cancer cell itself or soluble mucins produced by the cancer cell [13].

Serum AFP levels increase by 20–80% in HCC patients and are strongly associated with tumor aggressiveness [19–21]. High level of AFP is correlated with tumor size, vascular invasion and poorly differentiated HCC [19,22,23]. In our analysis, we found that siglec-2 expression in tumor tissues was significantly negatively associated with AFP elevation. Although the immunogenicity of AFP is weak, it could induce the immune escapes through inhibiting the function of dendritic cells, natural killer cells and T lymphocytes [24,25]. Several studies demonstrated that AFP is involved in immunosuppression [25,26]. It can impair the function of macrophages leading to decreased phagocytosis and impaired antigen-presenting abilities [27]. AFP-modified immune cell vaccine or peptide vaccine has displayed the specific antitumor immunity against AFP-positive tumor cells [28,29]. Hence, siglec-2 could play antitumor effects via enhancing immune responses by inhibition AFP levels. Although the proportion of patients with elevated AFP in siglec-2 low expression group was significantly higher than that in siglec-2 high expression group (60.0% vs. 41.7%), the biologic value is not strong. Further research with larger samples are needed.

Our results also showed that siglec-2 elevation predicts better survival in HCC. Siglecs including siglec-2 have been reported to regulate cell growth and survival, by both inhibition of proliferation and/or induction of apoptosis [13]. Throughout the last decade, several novel therapeutic agents that target siglec-2 are being developed as an alternative approach for cancer treatment [17,18,30]. Previous reports showed that siglec-2 as a B-cell-associated adhesion protein appeared to play a critical role in establishing signaling thresholds for B-cell activation, mediating normal antibody response to thymus-independent antigens and regulating the lifespan of mature B cells [31,32]. Therefore, down-regulating of siglec-2 in tumor tissues might risk the tumor progress by reducing innate immune response and mature B cells proliferation in HCC patients. Recently, it is gradually recognized that some B-cell subpopulations including regulatory B cells can impair CD4^+^ T cell activation or produce cytokines promote tumor progression [33–35], Leading to dramatically suppress antibody and inhibit antitumor effector T cells [34,36]. Lymphotoxin secreted from tumor-infiltrating B cells also promotes tumor growth [37]. Therefore, serves as B cell receptor inhibitor, siglec-2 might suppress tumor progress and development, contributing to a prolonging survival in HCC patients. Additionally, we enriched coexpressed genes of siglec-2 and its functional pathways. Siglec-2 and its coexpressed genes participant in the tumor cell phenotype including cell cycle, spliceosome, DNA replication, ubiquitin mediated proteolysis, proteasome, mismatch repair and pathways in cancer like MAPK signaling pathway and calcium signaling pathway, which should be the main research directions of siglec-2 mechanism in HCC in future.

Although siglec-4 levels in tumor tissues might associate with HCC OS in our Cox regression analysis, no significance was found in log-rank methods. Known as myelin-associated glycoprotein (MAG), siglec-4 is selectively localized in periaxonal Schwann cell and oligodendroglial membranes of myelin sheaths [38] and plays a role in axon-myelin stabilization and inhabitation of axon regeneration after injury [39,40]. Since siglec-4 is only found in the nervous system, even though siglec-4 showed some significance for HCC OS in our analysis, deep research of this gene in HCC development should be cautious and well-designed.

The present study has some limitations: First, our research was a preliminary analysis from GEO database, no further mechanism data were shown. Second, we included siglecs as a continuous variable in the logistic and Cox regression process, leading to a small HRs of the siglecs biomarker candidates. Third, only siglec-1 to siglec-9 were included in this analysis, other siglec family members like siglec-10 to siglec-15 were not available in this gene database. Fourth, we did not conduct mechanism research in siglec-2 protein level. Even with these limitations, the results might provide useful insights for HCC research in therapeutic strategy.

## Abbreviations

AFP: alpha-fetoprotein
GEO: Gene Expression Omnibus
HBV: hepatitis B virus
HCC: hepatocellular carcinoma
OS: overall survival
siglec: sialic-acid-binding immunoglobulin-like lectin
